# Comparison of Accuracy of Current Ten Intraoral Scanners

**DOI:** 10.1155/2021/2673040

**Published:** 2021-09-13

**Authors:** Pokpong Amornvit, Dinesh Rokaya, Sasiwimol Sanohkan

**Affiliations:** ^1^Department of Prosthetic Dentistry, Faculty of Dentistry, Prince of Songkla University, Hat Yai, Songkhla 90110, Thailand; ^2^Department of Clinical Dentistry, Walailak University International College of Dentistry, Walailak University, Bangkok 10400, Thailand

## Abstract

There have been various developments in intraoral 3D scanning technology. This study is aimed at investigating the accuracy of 10 scanners developed from 2015 to 2020. A maxillary dental model with reference points was printed from Form 2 (FormLabs, Somerville, MA, USA). The model was scanned 5 times with each intraoral scanner (IOS); Trios 3 (normal and high-resolution mode); Trios 4 (normal and high-resolution mode) (3Shape Trios A/S, Copenhagen, Denmark); iTero Element, iTero 2, and iTero 5D Element (Align Technologies, San Jose, California, USA); Dental Wings (Dental Wings, Montreal QC, Canada); Panda 2 (Pengtum Technologies, Shanghai, China); Medit i500 (Medit Corp. Seoul, South Korea); Planmeca Emerald™ (Planmeca, Helsinki, Finland); and Aoralscan (Shining 3D Tech. Co., Ltd., Hangzhou, China). After the scan, the 3D scanned stereolithography files were created. The various distances were measured five times in *X*, *Y*, *Z*, and *XY* axes of various scans and with a vernier caliper (control) and from the Rhinoceros software. The data were analyzed using SPSS 18. Test for the normality of the various measurement data were done using Kolmogorov-Smirnov test. The trueness and precision of the measurements were compared among the various scans using the Kruskal-Wallis test. The significance was considered at *P* < 0.05. The trueness of the intraoral scans was analyzed by comparing the measurements from the control. Precision was tested through the measurements of repeated scans. It showed that more the distance is less the accuracy for all scanners. In all studied scanners, the trueness varied but precision was favorably similar. Diagonal scanning showed less accuracy for all the scanners. Hence, when scanning the full arch, the dentist needs to take more caution and good scan pattern. Trios series showed the best scan results compared to other scanners.

## 1. Introduction

In recent decades, there has continuous advancement in digital technologies in dentistry, such as computer-aided design/computer-aided manufacturing (CAD/CAM) systems, milling systems, three-dimensional (3D) scanning, and printing of various dental biomaterials [1–3]. Digital dentistry helps in the diagnosis, treatment planning, and fabrication of prostheses. An accurate dental impression is required to fabricate a good dental prosthesis or restoration [4, 5]. To fabricate a prosthesis or restoration digitally, dentists send the digital impression obtained from an intraoral scanner (IOS) from the clinic to the dental laboratory. Then, after receiving the digital scan, the dental technician creates a digital model, then designs, and finally manufactures the prosthesis.

There are different IOSs that are available in the market [6]. Intraoral scanners generally have a scan area of 1-2 teeth [7, 8]. At present, there are advanced scanning technologies, such as triangulation technique (used by Cerec, Dentsply Sirona), active wavefront sampling (used by True Definition, 3 M ESPE), and confocal scanning technique (used by iTero, Align Technology, and Trios, 3Shape) [9–11]. The confocal scanning technology is a faster scanning technology that captures images by focusing on an optical light beam with high-resolution visual images with improved accuracy and fewer distortions [9, 12].

Hence, with the various developments in intraoral 3D scanning technology, it is important to access the scanning accuracy of various IOS in the market. Hence, this in vitro study is aimed at investigating the accuracy of 10 scanners developed from 2015 to 2020.

## 2. Materials and Methods

### 2.1. Study Model

Maxillary dental models with reference point model were drawn by CAD software using Meshmixer and were printed from Form 2 (Figure 1) (FormLabs, Somerville, MA, USA) [13, 14].

### 2.2. Scanning and 3D Model

The model was scanned 5 times with each intraoral scanner (IOS); Trios 3 (normal and high-resolution mode); Trios 4 (normal and high-resolution mode) (3Shape Trios A/S 2020, Copenhagen, Denmark); iTero Element, iTero 2, and iTero 5D Element (Align Technologies, San Jose, California, USA);Dental Wings (DentalWings, Montreal QC, Canada); Panda (Pengtum Technologies, Shanghai, China); Medit i500 (Medit Corp. Seoul, South Korea), Planmeca Emerald™ (Planmeca, Helsinki, Finland); and Aoralscan (Shining 3D Tech. Co., Ltd. Hangzhou, China) (Figure 2). Then, the 3D scanned files were saved as stereolithography (.STL).

### 2.3. Measurements

The various distances were measured five times in *X*, *Y*, *Z*, and *XY* (Figure 3). The *XY* represented the measurement crossing the midline, and we designated it as diagonal. The measurements were measured from the Rhinoceros software (Rhino, Robert McNeel & Associates, Washington DC, USA). Measurements measured from a vernier caliper were used as the control.

### 2.4. Statistical Analysis

The data were analyzed using SPSS 18. Test for the normality of the various measurement data were done using Kolmogorov-Smirnov test. The trueness and precision of the measurements were compared among the various scans using the Kruskal-Wallis test. The significance was considered at *P* < 0.05. The trueness of the intraoral scans was analyzed by comparing the measurements from the control. Precision was tested through the measurements of repeated scans.

## 3. Results

The results of various measurements in *X*, *Y*, *XY*, and diagonal measurements are shown in Tables 1–4.  Table 5 shows the results of the test for the normality of data using Kolmogorov-Smirnov of various measurements. It showed that the data are not normally distributed. It showed that there was a significant difference for all the measurements among the scanners. In all studied scanners, the trueness varied but precision was favorably similar.

It showed that the more the distance, the less is the trueness. For the precision, there was no significant difference (*P* > 0.05) from the Kruskal-Wallis test. For scanning in the diagonal axis, there was less accuracy for all scanners. Trios series showed better trueness and precision results compared to other scanners.

The mean difference of the various measurements of different IOS in various axes is shown in Figures 4–7.

## 4. Discussion

The IOS has various advantages such as they make easier for the clinician and the laboratory technicians to communicate, eliminating the dental plaster models and reduce the working time. The precision and trueness of the IOS are an important factor as it influences the restorations [1, 2].

In this study, the accuracy of various scans is studied. The surface area in the *X*-axis and *Y*-axis ranged from 2 to 60 mm The accuracy of scans followed *Y* − axis > *X* − axis = *Z* − axis > diagonal axis. In the posterior area, the accuracy is more, whereas in the anterior area, the accuracy is less as the shape of teeth creates more error when capturing the images. The scanning depth (*Z*-axis) ranged from 2 to 8 mm, where special precaution is needed especially in the deep cavity.

A study by Mutwalli et al. [15] found that regarding the interarch distance measurements, Trios 3 had the lowest trueness, followed by Trios 3 mono and Itero Element, But Trios had the lowest precision, followed by iTero Element and Trios 3 Mono. But in our study, the Trios series presented higher accuracy compared to other IOS. Our study is supported by another study done by Renne et al. [8] where they found that for complete-arch scanning, the 3Shape Trios was found to have the best balance of speed and accuracy.

The result of our study is supported by the study done by Medina-Sotomayor et al. [16] where they compared the scanning strategy with the greatest accuracy, in terms of trueness and precision, of 4 IOS in the impression of a complete dental arch. They found that the trueness of the Trios and iTero system showed better results with strategy “D,” Omnicam with strategy “B,” and True Definition with strategy “C.” In terms of precision, both iTero and True Definition showed better results with strategy “D,” while Trios showed the best results with strategy “A” and Omnicam with strategy “B.” There were significant differences between the scanning strategies with the iTero scanner, but not with the other scanners. They concluded that the digital impression systems used in the experiment provided sufficient flexibility for the acquisition of 3D images without this affecting the accuracy of the scanner.

Similarly, another study [17] evaluated the trueness and precision of 2 widely used intraoral scanners (Trios 3, 3Shape, and CS 3600, Carestream), using an industrial scanner (Artec Space Spider) as a reference. Surface-based matching was implemented using the iterative closest point algorithm (ICP). Trios 3 showed slightly higher precision (approximately 10 *μ*m) compared to CS 3600, only after superimposition on the whole dental arch (*P* < 0.05). Both intraoral scanners showed good performance and comparable trueness. However, in individual cases and various, not spatially defined areas, higher imprecision was evident. Thus, the IOS appropriateness for highly demanding, spatially extended clinical applications remains questionable.

Errors can occur which scanning by the IOS. The IOS captures approx. 1200 images when scanning. Scanning errors can result from the superimposition of the images while scanning and processing [7, 8]. This is due to the deviations of images which are more seen in the anterior teeth which have steep inclines and less tooth surface. Errors also can occur while computer processing from filter algorithms and calibration [18, 19]. In addition, errors during computer processing are due to filter algorithms [7]. Errors can occur on any axis. In this study, more errors were seen while scanning the depth (*Z*-axis).

Other factors that can affect the accuracy of IOS are intraoral factors (temperature, relative humidity, and illumination), operator (scanning pattern and skill), scanner unit (capture box, receiver, light source), computer software speed, and scanning area (scanning area, length, and surface irregularities) [20–23]. These factors were not considered in this study. In addition, since the model in this study overlaps the tooth with a complex shape, the side of these rectangular parallelepipeds can be scanned only when the scanner is tilted more. It is thought to be different from the usual scanning strategy performed in the actual clinical setting.

## 5. Conclusion

Within the limitations of this study, the following conclusions can be drawn.

1. More the scan distance, less the accuracy for all the scanners
2. In all studied scanners, the trueness varied but precision was favorably similar
3. Diagonal scanning showed less accuracy for all the scanners. Hence, when scanning the full arch, the dentist needs to take more caution and good scan pattern
4. Trios series showed the best scan results compared to other scanners

## Figures and Tables

**Figure 1:** 3D model. (a) The model was drawn by CAD software using Meshmixer, (b) 3D printed model, and (c) scanned file from an intraoral scanner exported to Rhinoceros 3D modeling software for the measurements.

**Figure 2:** Various scanners used in this study: (a) Trios 3, (b) Trios 4, (c) iTero Element, (d) iTero 2, (e) iTero 5D Element, (f) Dental Wings, (g) Panda, (h) Medit i500, (i) Planmeca Emerald™, and (j) Aoralscan.

**Figure 3:** Various measurements in *X*, *Y*, and *X*-axis.

**Figure 4:** Mean difference of the various measurements of different intraoral scanners in *X-*axis.

**Figure 5:** Mean difference of the various measurements of different intraoral scanners in *Y-*axis.

**Figure 6:** Mean difference of the various measurements of different intraoral scanners in the *Z*-axis.

**Figure 7:** Mean difference of the various measurements of different intraoral scanners in *XY* axis (diagonal).

**Table 1:** Results of measurements in *X*-axis measured from various scanners.

	Control	A (*N*)	A (HD)	A (*N*)	B (HD)	C	D	E	F	G	H	I	J
*X*1	1.90 ± 0.03	1.87 ± 0.03	1.88 ± 0.03	1.93 ± 0.04	1.88 ± 0.01	1.78 ± 0.032	1.80 ± 0.09	1.82 ± 0.07	1.87 ± 0.05	1.90 ± 0.03	1.80 ± 0.07	1.95 ± 0.02	1.87 ± 0.06
*X*2	9.92 ± 0.02	9.86 ± 0.03	9.96 ± 0.02	9.89 ± 0.03	9.87 ± 0.02	9.86 ± 0.02	9.89 ± 0.06	9.87 ± 0.06	9.86 ± 0.07	9.92 ± 0.02	9.77 ± 0.6	9.96 ± 0.08	9.92 ± 0.04
*X*3	29.84 ± 0.05	29.73 ± 0.02	29.91 ± 0.03	29.87 ± 0.07	29.82 ± 0.02	29.77 ± 0.05	29.71 ± 0.14	29.75 ± 0.07	29.80 ± 0.17	29.84 ± 0.05	29.55 ± 0.11	29.76 ± 0.73	29.83 ± 0.06
*X*4	39.89 ± 0.04	39.71 ± 0.01	39.69 ± 0.24	39.97 ± 0.06	39.97 ± 0.03	39.73 ± 0.10	40.74 ± 0.18	39.80 ± 0.06	39.11 ± 0.17	39.89 ± 0.04	39.58 ± 0.08	39.70 ± 0.28	39.94 ± 0.03
*X*5	50.01 ± 0.02	49.86 ± 0.11	50.21 ± 0.13	50.15 ± 0.03	50.14 ± 0.04	50.06 ± 0.08	49.87 ± 0.20	50.09 ± 0.20	50.83 ± 0.42	50.01 ± 0.02	49.61 ± 0.15	50.04 ± 0.23	50.33 ± 0.06
*X*6	60.53 ± 0.05	60.06 ± 0.27	60.36 ± 0.51	60.53 ± 0.13	60.64 ± 0.23	61.60 ± 0.08	61.53 ± 0.33	61.56 ± 0.14	61.95 ± 0.37	61.74 ± 0.24	61.58 ± 0.33	61.51 ± 0.33	61.51 ± 0.15

A (*N*): Trios3 (normal); A (HD): Trios3HR; B (*N*): T rios4; B (HD): Trios4HR; C: iTero Element; D: iTero Element2; E: iTero Element 5D; F: Dental Wings; G: Panda; H: Planmeca Medit i500; I: Emerald™; J: Aoralscan.

**Table 2:** Results of measurements in *Y*-axis measured from various scanners.

	Control	A (*N*)	A (HD)	A (*N*)	B (HD)	C	D	E	F	G	H	I	J
*Y*1	1.92 ± 0.15	1.85 ± 0.03	1.85 ± 0.07	1.91 ± 0.04	1.86 ± 0.02	1.71 ± 0.09	1.87 ± 0.17	1.81 ± 0.12	1.82 ± 0.01	1.92 ± 0.01	1.77 ± 0.02	1.87 ± .0.09	1.80 ± 0.03
*Y*2	9.87 ± 0.02	9.98 ± 0.14	9.81 ± 0.82	9.91 ± 0.06	9.84 ± 0.33	9.68 ± 0.98	9.78 ± 0.17	9.72 ± 0.06	9.80 ± 0.07	9.87 ± 0.02	9.73 ± 0.10	9.72 ± 0.13	9.90 ± 0.04
*Y*3	19.80 ± 0.37	19.71 ± 0.12	19.81 ± 0.06	19.83 ± 0.04	19.83 ± 0.08	19.57 ± 0.09	19.74 ± 0.19	19.50 ± 0.24	19.63 ± 0.51	19.80 ± 0.03	19.67 ± 0.10	19.50 ± 0.01	19.76 ± 0.12
*Y*4	30.47 ± 0.16	29.97 ± 0.39	30.18 ± 0.59	29.69 ± 0.13	29.63 ± 0.07	29.47 ± 0.13	29.48 ± 0.33	29.49 ± 0.42	29.75 ± 0.42	29.47 ± 0.37	29.47 ± 0.03	29.41 ± 0.09	29.77 ± 0.29

A (*N*): Trios3 (normal); A (HD): Trios3HR; B (*N*): Trios4; B (HD): Trios4HR; C: iTero Element; D: iTero Element2; E: iTero Element 5D; F: Dental Wings; G: Panda; H: Planmeca Medit i500; I: Emerald™; J: Aoralscan.

**Table 3:** Results of measurements in *Z*-axis measured from various scanners.

	Control	A (*N*)	A (HD)	A (*N*)	B (HD)	C	D	E	F	G	H	I	J
*Z*1	2.00 ± 0.17	2.01 ± 0.03	1.99 ± 0.04	1.99 ± 0.04	1.97 ± 0.02	1.92 ± 0.02	1.99 ± 0.08	1.91 ± 0.07	1.99 ± 0.06	2.00 ± 0.17	1.89 ± 0.06	1.88 ± 0.11	1.95 ± 0.03
*Z*2	3.98 ± 0.01	3.98 ± 0.07	3.95 ± 0.07	4.00 ± 0.04	3.98 ± 0.02	3.94 ± 0.02	3.82 ± 0.09	3.91 ± 0.15	3.97 ± 0.05	3.98 ± 0.01	3.94 ± 0.08	3.80 ± 0.14	4.00 ± 0.06
*Z*3	6.08 ± 0.03	5.90 ± 0.20	5.97 ± 0.01	5.99 ± 0.04	5.95 ± 0.04	5.83 ± 0.13	5.85 ± 0.06	5.81 ± 0.16	6.14 ± 0.15	6.08 ± 0.03	5.87 ± 0.07	5.85 ± 0.04	5.89 ± 0.07
*Z*4	8.12 ± 0.08	7.96 ± 0.08	7.97 ± 0.13	7.93 ± 0.05	7.96 ± 0.03	7.83 ± 0.05	7.83 ± 0.10	7.71 ± 0.34	7.99 ± 0.15	8.12 ± 0.08	7.92 ± 0.13	7.83 ± 0.06	7.91 ± 0.13

A (*N*): Trios3 (Normal); A (HD): Trios3HR; B (*N*): Trios4; B (HD): Trios4HR; C: iTero Element; D: iTero Element2; E: iTero Element 5D; F: Dental Wings; G: Panda; H: Planmeca Medit i500; I: Emerald™; J: Aoralscan.

**Table 4:** Results of measurements in diagonal measured from various scanners.

	Control	A (N)	A (HD)	A (N)	B (HD)	C	D	E	F	G	H	I	J
AR	65.06 ± 0.03	64.87 ± 0.11	65.12 ± 0.17	64.83 ± 0.47	65.08 ± 0.46	66.42 ± 0.38	66.48 ± 0.55	66.41 ± 0.44	66.44 ± 0.26	66.43 ± 0.33	66.46 ± 0.32	66.49 ± 0.30	66.52 ± 0.39
AL	65.32 ± 0.60	65.43 ± 0.48	65.40 ± 0.32	65.28 ± 0.13	65.27 ± 0.13	66.56 ± 0.17	66.55 ± 0.48	66.62 ± 0.25	66.56 ± 0.41	66.81 ± 0.44	66.63 ± 0.45	66.71 ± 0.48	66.64 ± 0.07

A (*N*): Trios3 (Normal); A (HD): Trios3HR; B (*N*): Trios4; B (HD): Trios4HR; C: iTero Element; D: iTero Element2; E: iTero Element 5D; F: Dental Wings; G: Panda; H: Planmeca Medit i500; I: Emerald™; J: Aoralscan.

**Table 5:** The results of the test for normality of data using Kolmogorov-Smirnov of various measurements.

Various measurements	Kolmogorov-Smirnov^a^		
	Statistic	Degree of freedom	*P* value
*X*1	0.120	65	0.022^∗^
*X*2	0.104	65	0.076^∗^
*X*3	0.097	65	0.200^∗^
*X*4	0.127	65	0.011^∗^
*X*5	0.125	65	0.013^∗^
*X*6	0.147	65	0.001^∗^
*Y*1	0.072	65	0.200^∗^
*Y*2	0.130	65	0.008^∗^
*Y*3	0.146	65	0.001^∗^
*Y*4	0.152	65	0.001^∗^
AR	0.164	65	<0.0001^∗^
AL	0.172	65	<0.0001^∗^
*Z*1	0.181	65	<0.0001^∗^
*Z*2	0.139	65	0.003^∗^
*Z*3	0.056	65	0.200^∗^
*Z*4	0.085	65	0.200^∗^

^a^Lilliefors Significance Correction; ^∗^significant at *P* value <0.05.

## Data Availability

The data used to support the findings of this study are available from the corresponding author upon reasonable request.
